The article "Serotonin Regulates the Firing of Principal Cells of the Subiculum by Inhibiting a T-type Ca2+ Current" was published in 2017. Journal: Front Cell Neurosci.

# Serotonin Regulates the Firing of Principal Cells of the Subiculum by Inhibiting a T-type Ca^2+^ Current

**DOI:** 10.3389/fncel.2017.00060

**Published:** 2017-03-07

**Authors:** Anders V. Petersen, Camilla S. Jensen, Valérie Crépel, Mathias Falkerslev, Jean-François Perrier

**Affiliations:** ^1^Department of Neuroscience and Pharmacology, University of CopenhagenCopenhagen, Denmark; ^2^Department of Biomedical Sciences, University of CopenhagenCopenhagen, Denmark; ^3^Institut de Neurobiologie de la Méditerranée (INMED), Institut National de la Santé et de la Recherche Médicale (INSERM) U901, Aix-Marseille UniversitéMarseille, France

**Keywords:** serotonin, subiculum, calcium channels, burst firing, temporal lobe epilepsy (TLE)

## Abstract

The subiculum is the main output of the hippocampal formation. A high proportion of its principal neurons fire action potentials in bursts triggered by the activation of low threshold calcium currents. This firing pattern promotes synaptic release and regulates spike-timing-dependent plasticity. The subiculum receives a high density of fibers originating from the raphe nuclei, suggesting that serotonin (5-HT) modulates subicular neurons. Here we investigated if and how 5-HT modulates the firing pattern of bursting neurons. By combining electrophysiological analysis with pharmacology, optogenetics and calcium imaging, we demonstrate that 5-HT_2C_ receptors reduce bursting activity by inhibiting a low-threshold calcium current mediated by T-type Ca^2+^ channels in principal cells of the subiculum. In addition, we show that the activation of this novel pathway decreases bursting activity and the occurrence of epileptiform discharges induced in *in vitro* models for temporal lobe epilepsy (TLE).

## Introduction

The subiculum is the major output of hippocampal formation. It relays information from and to CA1 hippocampal region, cortical (entorhinal, perirhinal, retrosplenial) and subcortical regions (mammillary nucleus, pre-subiculum, nucleus accumbens; Naber and Witter, 1998; O’Mara et al., 2001). Because of this central position, the subiculum plays important roles in diverse functions such as spatial navigation (Sharp and Green, 1994; O’Mara et al., 2000) or learning and memory (Morris et al., 1990; Galani et al., 1998). In addition the subiculum becomes a source for temporal lobe epilepsy (TLE) when its principal cells are hyperexcitable (Cohen et al., 2002; Wellmer et al., 2002; Wozny et al., 2005). Depending on the ion channels expressed in their membranes, pyramidal cells fire action potentials regularly or in bursts caused by the activation of transient calcium currents (Jung et al., 2001). These intrinsic properties are essential for synaptic integration, as notable differences have been reported for the processing of signals by the two types of neurons. Long-term potentiation (LTP) relies on an increase in calcium concentration for regular firing cells but not for bursting neurons (Wozny et al., 2008). In contrast, postsynaptic bursts induce long-term depression (LTD) when causally paired with EPSPs but induce LTP when anticausally paired (Pandey and Sikdar, 2014). The fine-tuning of bursting behavior could therefore have an important impact on spike-timing-dependent plasticity.

Pyramidal cells from the hippocampus are modulated by serotonin (5-HT) released into the extracellular space by *en passant* synapses (Andersen, 2007). Interestingly the density of serotonergic terminals is the highest in the subiculum (Oleskevich and Descarries, 1990), suggesting that the monoamine is a major modulator of principal neurons.

Here we investigated if and how 5-HT modulates the firing properties of bursting neurons from the subiculum. By combining local field potential (LFP) recordings, patch clamp recordings, pharmacology, calcium imaging and optogenetics, we found that the activation of 5-HT_2C_ receptors decreases bursting by selectively inhibiting T-type Ca^2+^ channels. In addition, we show that the activation of the pathway we uncovered decreases the occurrence of epileptiform discharges induced in two *in vitro* models for TLE.

## Materials and Methods

### Mouse Brain Slice Preparation

Experiments were performed on juvenile to adult C57BL/6 mice (P12–P30; Taconic, Denmark and Janvier, France) and from TPH2-ChR2-YFP mice (B6; SJL-Tg (Tph2-COP4^*^H13R/EYFP) 5Gfng/J, JAX stock #014555) of both sexes (8–10 weeks of age) for optogenetics. The surgical procedures complied with Danish legislation. This study was carried out in accordance with the recommendations of Department of Experimental Medicine of the University of Copenhagen. The protocol was approved by the Department of Experimental Medicine of the University of Copenhagen. Mice were killed by decapitation. The brain was transferred into a cooled solution of artificial cerebrospinal fluid (ACSF) containing (in mM): NaCl 125, KCl 2.5, NaHCO_3_ 26, CaCl_2_ 2, MgCl_2_ 1, NaH_2_PO_4_ 1.25, Glucose 25. Parasagittal slices (300 μm) were cut with a vibratome (Microm HM 650V with CU 65 cooling unit or Leica VT1200). The slices were transferred to a dual-superfusion holding chamber containing 35°C ACSF at a high flow rate (>2 ml/min) continuously bubbled. The slices were pre-incubated for at least 1 h before measurement.

### Electrophysiology

Visual patch-clamp recording was performed with an upright microscope (Olympus BX51WI). The recording chamber was continuously perfused with oxygenated ACSF. Glass pipettes pulled on a Puller (Sutter Instruments P87; Novato, CA, USA) were filled with the following solution: (in mM) K-gluconate 122, Na_2_-ATP 5, MgCl_2_ 2.5, CaCl_2_ 0.0003, Mg-Gluconate 5.6, K-Hepes 5, H-Hepes 5, EGTA 1 (all from Sigma-Aldrich), Biocytin 10 (Invitrogen), Alexa Fluor 488 Hydrazide 1 (Invitrogen). KOH was added to adjust the pH at 7.3–7.4. Recordings were performed in whole-cell configuration. The recording electrodes (resistance 4–6 MΩ) were mounted on micromanipulators (Luigs and Neumann, Germany) and connected to CV-7B Current-Clamp and Voltage-Clamp Headstages (Molecular Devices, Sunnyvale, CA, USA). Recordings were acquired with a Multiclamp 700B amplifier and Digidata 1322A or 1440A Digitizer.

### Induction of Epileptiform Discharges

Epileptiform activity was induced by applying an ACSF where MgCl_2_ was replaced by CaCl_2_. LFP were recorded in the subiculum with glass electrodes (2–3 MΩ; filled with normal ACSF). Epileptiform discharges were evoked by stimulation performed with a bipolar concentric electrode (TM33CCNON; World Precision Instruments, Sarasota, FL, USA) connected to an isolation unit (Isolator 11, Axon Instruments, Union City, CA, USA) triggered by an external signal. The stimulation electrode was positioned in the *stratum oriens* and *alveus* of CA1.

### Calcium Imaging

Calcium imaging of individual cells was obtained by adding the Ca^2+^ sensitive dye Fura-2 (200 μM; Invitrogen) to the patch solution. The dye was excited at 340 nm with a monochromator (Till Photonics, Germany). The fluorescence was measured through an emission filter at 510 nm with a digital camera (QImaging Retiga-2000RV Camera) controlled by Till Vision software (v.4.0.1). Frames were collected every 399 ms.

### Pharmacology

Neurons were isolated from their surrounding synaptic environment by blocking AMPA, NMDA and GABA_A_ and glycine receptors with CNQX (20 μM, Tocris), AP5 (50 μM, Tocris), Gabazine (10 μM, Tocris) and Strychnine (10 μM, Sigma-Aldrich). Ca^2+^ currents were isolated by blocking voltage gated K^+^ channels with 4-Aminopyridine (4-AP, 3 mM; Sigma-Aldrich), tetraethylammonium (TEA, 0.1 mM; Sigma-Aldrich) cesium (1 mM; Sigma-Aldrich) and Na^+^ channels with tetrodotoxin (TTX, 1 μM; Alomone Labs). Drugs applied to the extracellular medium: 5-HT hydrochloride (10 μM; Sigma Aldrich); 4-Iodo-2,5-dimethoxy-α-methylbenzeneethanamine hydrochloride (DOI hydrochloride; 10–20 μM, Tocris); Mibefradil (8–16 μM, Tocris).

### Focal Application of Drugs

Focal application of drugs was obtained with a glass pipette (diameter 2–3 μm) mounted on a micromanipulator. Drugs: 8,9-Dichloro-2,3,4,4a-tetrahydro-1*H*-pyrazino[1,2-*a*]quinoxalin-5(6*H*)-one hydrochloride (WAY 161503 hydrochloride; 500 μM, Tocris), 1,2,3,4,8,9,10,11-Octahydro[1,4]diazepino[6,7,1-*jk*]carbazole hydrochloride (WAY 629 hydrochloride; 10 μM, Tocris), 5-HT hydrochloride (1.5 mM; Sigma Aldrich). 5-HT was also applied by means of microiontophoresis. Glass micropipettes were filled with 5-HT hydrochloride (100 mM; pH 4). Diffusion of 5-HT from the pipette was minimized by a holding current of −50 nA. 5-HT was released by positive current pulses (10–150 nA; 1–5 s).

### Immunohistochemistry and Imaging

Slices were fixed in 4% paraformaldehyde in PBS for 30 min at 4°C before staining. Free-floating slices were washed in PBS and permeabilized overnight at 4°C with 1% triton X-100 dissolved in PBS. The slices were blocked for 3 h in blocking buffer (4% milk, 0.3% Triton X-100/PBS), stained with primary antibodies diluted in blocking buffer (2–3 days at 4°C) and washed in PBS. Immunoreactivity was detected using Alexa dye-conjugated secondary antibodies diluted in blocking buffer. The slices were incubated with the secondary antibodies for 2 h and then washed in 0.1% triton X-100 in PBS. Finally, slices were washed 2–3 times in PBS and mounted with ProLong Gold antifade reagent (Life Technologies) on glass microscope slides. Imaging was performed with Zeiss LSM 780 confocal system equipped with a 20× (LD Plan Neofluar, NA 0.8) and a 63× (Plan Apochromat, NA 1.4) oil immersion objective with a pinhole size of one and pixel format of 1024 × 1024. Line averaging was performed to reduce noise. Images were transferred to ImageJ/FIJI.

### Antibodies and Dyes

Voltage-gated calcium channels were detected with rabbit polyclonal antibodies from Alomone (Ca_V_3.1:ACC-021 and Ca_V_3.3:ACC-009) in a concentration 1:50. 5-HT was detected with a rat monoclonal antibody (1:100; Milipore). 5-HT_2C_ receptors were detected by a mouse monoclonal IgG1 antibody (BD Pharmigen; clone SR-2C) in concentration 1:100. Microtubule associated protein 2 (MAP2) was detected with a mouse monoclonal IgG1 antibody (Sigma; clone HM-2) in concentration 1:300 or rabbit polyclonal IgG (Santa-Cruz, MAP-2 Antibody (H-300) in concentration 1:100), DAPI nucleic acid stain (1 mg/ml; Invitrogen D-9542) in concentration 1:300.

### Slice from the Hippocampus of Pilocarpine Treated Rats

All experiments were approved by the Institut National de la Santé et de la Recherche Médicale animal care and use agreement (D-13-055-19) and the European community council directive (2010/63/UE). Rats (5–6 weeks, 150–350 g, Janvier, France) were injected intraperitoneally with pilocarpine hydrochloride (340 mg/kg) 30 min after the peripheral cholinergic antagonist scopolamine methyl nitrate (1 mg/kg, i.p.). Eighty percent of the rats experienced class IV/V seizures. After 2–3 h of *status epilepticus*, diazepam (8 mg/kg) was injected (i.p.). After a seizure-free period of several weeks, we selected for recordings and analysis only rats that experienced recurrent spontaneous seizures (7–11 months after the pilocarpine injection; *n* = 3). Rats were anesthetized with chloral hydrate (70 mg/kg, i.p.) and decapitated. The brain was removed, the hippocampi were dissected, and transverse 400 μm-thick hippocampal slices were cut with a Leica VT1000S tissue slicer (Leica, Germany) in a solution containing the following (in mM): 132.5 choline chloride, 2.5 KCl, 1.25 NaH_2_PO_4_, 26 NaHCO_3_, 7 MgCl_2_, 0.5 CaCl_2_, and 7 D-glucose (2–5°C). Slices were then transferred for rest at room temperature (>1 h) in oxygenated normal ACSF containing the following (in mM): 126 NaCl, 3.5 KCl, 1.2 NaH_2_PO_4_, 26 NaHCO_3_, 1.3 MgCl_2_, 2.0 CaCl_2_, and 10 D-glucose, pH 7.4. This solution is referred to as rat ACSF (rACSF). Acute slices were transferred to a recording chamber maintained at 30–32°C and perfused (2 ml/min) with oxygenated normal ACSF. LFP were recorded in the subiculum with glass electrodes (2–3 MΩ; filled with normal ACSF) using a DAM-80 amplifier (bandpass filter, 1–3 Hz; World Precision Instruments, Sarasota, FL, USA) and evoked by electrical stimulations with bipolar NiCh electrodes (NI-0.7F, Phymep, France) positioned in the *stratum oriens* and *alveus* of CA1.

### Data Analysis

Data were analyzed with Clampfit 10 (Molecular Devices), Matlab (Mathworks) and GraphPad Prism. Samples were compared by non-parametric tests. Data are represented as mean ± standard deviation (SD) or standard error of the mean (SEM), as stated in the text. Statistical significance was assessed by non-parametric Wilcoxon signed-rank test and kolmogorov-smirnov two sample test, *P < 0.05, **P < 0.01, ***P < 0.001.

## Results

### Serotonin Inhibits the Burst Firing of Pyramidal Neurons from the Subiculum

We characterized the firing behavior of principal cells from the subiculum by recording the electrical activity of individual pyramidal cells using patch-clamp technique, LFP, optogenetics and calcium imaging. In agreement with previous observations (Mason, 1993; Stewart and Wong, 1993; Taube, 1993), we found that 284 out of 351 (81%) pyramidal cells recorded in the distal half of the subiculum, responded to depolarizing current pulses with a burst of action potentials followed by regular firing (Figure 1A; mice age P12–P28). The probability of generating a burst was increased when evoked from a hyperpolarized membrane potential and decreased when evoked from a depolarized membrane potential (Figure 1B), suggesting involvement of a voltage-sensitive conductance partly de-inactivated at rest and sharing the properties of T-type Ca^2+^ channels (Llinás and Yarom, 1981).

**Figure 1:** **Serotonin (5-HT) inhibits the bursting of principal cells from the subiculum. (A)** Response of a pyramidal cell to a depolarizing current pulse. **(B)** Burst probability as function of Vm. Only bursting cells are used for this plot. Hyperpolarization increased burst probability (*n* = 148). Blue: distribution of resting membrane potentials. **(C)** Response of the same cell as in **(A)** to the same depolarizing current pulse after a puff of 5-HT. **(D)** Decrease in number of spikes and membrane potential (−0.82 ± 1.29 tested 15 s after puffing 5-HT); *n* = 51; Wilcoxon test; hyperpolarization of −1.47 ± 1.43 mV; *n* = 51; Wilcoxon test. **(E)** Response of a yellow fluorescent protein (YFP+) neuron from the dorsal raphe nucleus of a tryptophan hydroxylase 2 (TPH2)-channelrhodopsin2 (ChR2)-YFP mouse to 480 nm light pulses. **(F)** Response of a pyramidal cell from the same mouse to a depolarizing pulse in control conditions and after 480 nm light pulses. **(G)** Mean number of spikes generated by pulses before and after light application. Significant decrease (Kolmogorov-Smirnov test; *n* = 3). **(H)** Black: response of pyramidal neuron from the subiculum to a hyperpolarizing followed by a depolarizing pulse. Red: 5-HT puff inhibited the burst. Inset: number of spikes in control and after puffing 5-HT. Significant decrease; Kolmogorov-Smirnov test (*n* = 11). **(I)** Ca^2+^ imaging obtained in the same neuron. Upper panels: Ca^2+^ signal increased during the burst. Plot, black: variations in Ca^2+^ concentration. Significant increase during the burst (from 0.02% to 0.44%; Kolmogorov-Smirnov test, *n* = 11). Red: after puffing 5-HT, the Ca^2+^ signal did not increase (ns: *p* = 0.14, Kolmogorov-Smirnov test, *n* = 11 cells, frame 1–4 vs. 7–9). Ca^2+^ signal significantly different from control conditions, Wilcoxon test (*n* = 11). **(J)** Left bar plot: example of cells for which 5-HT did not change the input resistance (Control 194.5 ± 15.98 MΩ SEM; 5-HT: 193.2 ± 17.63 MΩ, no significant decrease, *p* = 0.547, Wilcoxon signed rank test, *n* = 8). Right bar plot: number of spikes/burst for the same cells in control and after 5-HT (control: 3 ± 0.57 SEM, 5-HT: 0.88 ± 0.48 SEM, significant decrease, *p* = 0.0312; Wilcoxon signed rank test, *n* = 8). ^*^p < 0.05; ^*^^*^p < 0.01; ^*^^*^^*^p < 0.001.

Next, we tested how 5-HT modulated the electrical properties of principal cells. When 5-HT was puff-applied near the membrane, the number of spikes present in each burst decreased significantly (Figure 1C) and the membrane was slightly hyperpolarized (Figure 1D). Both effects were still present 15 s after the puff of 5-HT and developed with similar time courses (Figure 1D). The inhibition of the burst did not depend on changes in input resistance induced by 5-HT (Figure 1J; Significant decrease of bursts in cells with no decrease in input resistance: control input resistance 194.5 ± 15.98 MΩ SEM; 5-HT: 193.2 ± 17.63 MΩ, *p* = 0.547; Number of spikes/burst in control: 3 ± 0.57, 5-HT: 0.88 ± 0.48 SEM, *p* = 0.0312; Wilcoxon signed rank test, *n* = 8). We tested if synaptic release of 5-HT also inhibited the bursting with a mouse expressing channelrhodopsin2 (ChR2) and Yellow Fluorescent Protein (YFP) under the control of tryptophan hydroxylase 2 (TPH2; Zhao et al., 2011). Pulses of blue light triggered action potentials in YFP+ cells from raphe nuclei recorded in a slice preparation from the brainstem (*n* = 2; Figure 1E). In brain slices, bursts of action potentials evoked by depolarizing current pulses in principal cells from the subiculum were significantly inhibited by blue light acting on serotonergic terminals (Figures 1F,G; *n* = 3; mice age: 9 weeks). This observation suggests that synaptic release of 5-HT inhibited bursting activity. Since T-type Ca^2+^ channels trigger voltage-dependent bursts of action potentials (Llinás and Yarom, 1981), we checked if the intracellular Ca^2+^ concentration increased during bursts. After loading pyramidal cells with the Ca^2+^ indicator Fura-2, we monitored the fluorescence signal at 340 nm. The fluorescence intensity increased significantly during burst, suggesting an elevation of the intracellular free Ca^2+^ (Figures 1H,I; mice age P12–P28). When 5-HT was puff applied near the membrane, the burst was inhibited (Figure 1H) and the Ca^2+^ signal was attenuated (Figure 1I). Taken together, our results suggest that the activation of 5-HT receptors decreases bursting in principal cells by inhibiting T-type Ca^2+^ channels.

### Serotonin Inhibits Ca_V_3 Channels in Subicular Pyramidal Neurons

To test our hypothesis, we isolated Ca^2+^ currents by blocking Na^+^ conductances with TTX and K^+^ channels with a mixture of TEA, 4-AP and cesium. An activation protocol with a pre-hyperpolarization step, evoked a transient inward current (Figure 2A; mice age P14–P27) with a threshold around −50 mV. The current displayed large overlap between curves describing activation (data not shown), a characteristic found for T but not R-type Ca^2+^ channels (Randall and Tsien, 1997). Both the activation and the inactivation characteristics matched the properties of low-threshold T-type Ca^2+^ channels recorded in hippocampal neurons (Toselli and Taglietti, 1992; Figure 2B). Puff-application of 5-HT significantly decreased the amplitude of the current at all potentials held above the threshold for low threshold Ca^2+^ spikes (LTS; Figures 2A,C,D). Upon addition of mibefradil, most of the T-type calcium current was blocked (Figure 2C) and the inhibitory effect of 5-HT on the Ca^2+^ current was strongly reduced (Figures 2C,D). The current modulated by 5-HT was significantly inhibited by mibefradil (Figure 2D). The hyperpolarization induced by 5-HT could be caused by the inhibition of a window current mediated by T-type Ca^2+^ channels as described in other parts of the brain (Dreyfus et al., 2010). In agreement, we found that the negative current holding the membrane at −70 mV was reduced after puffing 5-HT (Figure 2E). In the presence of mibefradil, 5-HT still produced an inhibition of the inward current, but to a much lesser extent (Figures 2E,F). This suggests, that most of the hyperpolarization induced by 5-HT was mediated by the inhibition of a T-type window current. We verified that subicular neurons express T-type Ca^2+^ channels by means of immunohistochemical staining performed with antibodies directed against Ca_V_3.1, Ca_V_3.2 and Ca_V_3.3 subunits. We found expression of Ca_V_3.1 and Ca_V_3.3 on the soma and apical dendrites of pyramidal cells (Figures 2G,H), while Ca_V_3.2 staining was inconclusive (Data not shown). In addition, staining performed with an antibody directed against 5-HT revealed a dense innervation of the subiculum (Figure 2I). Altogether our data show that 5-HT decreases the burst firing of subicular neurons by inhibiting a current mediated by T-type Ca^2+^ channels.

**Figure 2:** **5-HT inhibits T-type Ca^2+^ current in pyramidal cells from the subiculum. (A)** Ca^2+^ current isolated by adding tetrodotoxin (TTX; 1 μM), tetraethylammonium (TEA; 0.1 mM), 4-Aminopyridine (4-AP; 3 mM) and cesium (1 mM). A depolarizing step from −85 mV to −35 mV evoked a transient low-threshold inward current (black). After puffing 5-HT, the amplitude of the current was decreased. Scale bars; 200 pA and 100 ms. **(B)** Normalized amplitude of the mean current (± SD) evoked during activation and inactivation protocols (insets). **(C)** Normalized amplitude of the current evoked during activation protocols in control conditions (black) and in mibefradil (8 μM; gray). Significant decrease (gray); Wilcoxon test (*n* = 10). Red: after puffing 5-HT in normal Ringer. Significant decrease (red stars); Wilcoxon test; *n* = 10. Orange: in mibefradil (8 μM), after puffing 5-HT (inhibition of 38.15% ± 61.20; Wilcoxon test; *n* = 10). **(D)** Normalized amplitude of current modulated by 5-HT (control—5-HT) in normal Ringer (red) and in mibefradil (orange). Significant inhibition (Wilcoxon test; *n* = 10). **(E)** Left: normalized holding current in control (black) and after 5-HT application (red); right: normalized holding current in mibefradil (8 μM; gray) before and after 5-HT application (orange). Error bars indicate SEM (Wilcoxon test; *n* = 10). **(F)** Average difference in holding current before and after 5-HT application in control conditions (red) and after mibefradil (8 μM; orange). Significant effect of mibefradil (Wilcoxon test; *n* = 10). **(G,H)** Immunohistochemical staining of the subiculum. Scale bar: 5 μm. Red: microtubule associated protein 2 (MAP2); Blue: DAPI; Green Ca_V_3.1 (g), Ca_V_3.3 (h). **(I)** Immunohistochemical staining of the subiculum. Scale bar: 100 μm. Green: 5-HT; Blue: DAPI. ^*^p < 0.05; ^*^^*^p < 0.01; ^*^^*^^*^p < 0.001.

### The Inhibition of T-type Channels Is Mediated by 5-HT_2C_ Receptors

Next we identified the serotonergic receptor responsible for the inhibition of T-type Ca^2+^ current. Similar to 5-HT, puff-application of the selective 5-HT_2C_ receptor agonists WAY 161503 or WAY 629 near the membrane decreased the number of spikes evoked during bursts of action potentials and hyperpolarized the membrane potential (Figures 3A,B; mice age P15–P19). Again, the inhibitory effect remained significant 15 s after applying the drug. The isolated Ca^2+^ current recorded in voltage-clamp mode was also significantly inhibited (Figures 3C,D). Our data suggest that 5-HT_2C_ receptors are responsible for the inhibition of T-type Ca^2+^ currents. We found that antibodies directed against 5-HT_2C_ receptors stained the dendrites of subicular pyramidal cells (Figure 3E) where Ca_V_3.1 and Ca_V_3.3 channels were also expressed (Figures 3F,G).

**Figure 3:** **5-HT_2C_ receptor activation inhibits T-channels in subicular pyramidal neurons. (A)** Response of a pyramidal cell to a depolarizing current pulse. The response consists of a burst (inset) followed by a train of action potentials. After puffing WAY 629 (10 μM), the burst was inhibited. Scale bars: 20 mV and 1 s. **(B)** Time course of the modulation induced by the 5-HT_2C_ receptor agonists WAY 161503 (500 μM) or WAY 629 (10 μM). Number of action potentials present in each burst decreased for more than 15 s, −1.81 ± 1.99 Wilcoxon test; *p* < 0.001 (*n* = 11) and the membrane hyperpolarized (−1.90 ± 1.12 mV when tested 10 s after drug application; Wilcoxon test; *n* = 12). **(C)** Voltage-clamp recording of the isolated Ca^2+^ current in control (black) and after puffing WAY 161503 (blue). Scale bars: 500 pA and 100 ms. **(D)** Normalized amplitude of the Ca^2+^ current as a function of V_h_ in control (black) and after puffing WAY 161503 (blue). Significant decrease (Wilcoxon test; *n* = 5). **(E–G)** Images of the subiculum. **(E)** 5-HT_2C_ receptors are expressed on dendrites identified with the marker MAP2. Upward arrows indicate positive staining for both 5-HT_2C_ receptors and MAP2. Downward arrows indicate MAP2 staining without 5-HT_2C_ receptors.** (F,G)** 5-HT_2C_ receptors expressed in the processes where Ca_V_3.1 and Ca_V_3.3 channels are found. Scale bar: 5 μm. ^*^p < 0.05; ^*^^*^p < 0.01; ^*^^*^^*^p < 0.001.

### Serotonin Decreases Epileptiform Discharges in the Subiculum

Subiculum is critical for seizure activity occurring in TLE in humans and rodents (Behr and Heinemann, 1996b; Cohen et al., 2002; Wozny et al., 2005). Under pathological conditions, the subicular pyramidal neurons that possess burst properties mediated by Ca^2+^ channels (Jung et al., 2001) lead the seizure activity (Menendez de la Prida and Gal, 2004). For these reasons, we evaluated the ability of 5-HT to prevent epileptiform discharges in the subiculum in slices from the hippocampus of pilocarpine treated chronic epileptic rats (see “Materials and Methods” Section). We recorded the electrical activity in the subiculum by means of a LFP electrode. A single electrical stimulation applied in *stratum oriens* and *stratum alveus* of CA1 evoked an epileptiform discharge including recurrent activities in normal rACSF (Figures 4A–D; *n* = 6 slices). This type of activity is never observed in normal animals when a single electrical stimulation is applied in normal rACSF (Taube, 1993; Colling et al., 1998; Wozny et al., 2008). In the presence of 5-HT (10 μM), the number of recurrent activities was strongly reduced (Figures 4A–D). This observation is in agreement with previous studies showing that 5-HT decreases the occurrence of seizures in the hippocampus (Prendiville and Gale, 1993; Yan et al., 1994; Bagdy et al., 2007; Buchanan et al., 2014). We obtained similar results in a slice preparation from the mouse brain with epileptiform activity induced by lowering the extracellular concentration of Mg^2+^ (Behr and Heinemann, 1996a; Harris and Stewart, 2001a; Menendez de la Prida and Gal, 2004). In this condition, spontaneous epileptiform events were present (Figure 4Q). Here again, a single shock applied in *stratum oriens* and *stratum alveus* of CA1 induced a barrage of recurrent activities in the subiculum (Figures 4E–H; mice age P15–P22). After addition of 5-HT (10 μM), the intensity of these activities was strongly decreased (Figures 4E–H; *n* = 8 slices) in accordance with previous studies (Behr and Heinemann, 1996a).

**Figure 4:** **5-HT inhibits evoked seizures in principal cells from the subiculum. (A)** Black: field recording from the subiculum in a brain slice from a pilocarpine treated rat. An electric shock applied in CA1 evoked recurrent bursts of activity. Red: in the presence of 5-HT (10 μM). Scale bars: 20 μV and 100 ms. **(B)** Time-frequency spectrograms of recurrent burst in control condition and in 5-HT. **(C)** Mean summed power spectrum analysis of recurrent bursts of the slice illustrated in **(A,B)**. Error bars: SD; Kolmogorov-Smirnov test; *n* = 30 sweeps. **(D)** Mean summed power spectrum of recurrent bursts in 5-HT as a function of the mean summed power in control conditions for the six slices tested. Error bars: SEM Reduction in the power spectrum from 50 Hz to 550 Hz of 23.84% ± 23.76%, Kolmogorov-Smirnov test. Significant decrease; Kolmogorov-Smirnov test; *n* = 6 slices and 30 recordings per slice. **(E)** Black: extracellular recording a pyramidal neuron from the subiculum recorded in a brain slice from a mouse after removal of extracellular Mg^2+^. Red: recording in 5-HT (10 μM). Bars: 10 mV and 100 ms. **(F)** Time-frequency spectrograms of recurrent burst in control condition and in the presence of 5-HT. **(G)** Mean summed power spectrum analysis of recurrent bursts of the slice illustrated in **(E,F)**. Kolmogorov-Smirnov test; *n* = 10 sweeps. **(H)** Mean summed power spectrum of recurrent bursts in 5-HT as a function of the mean summed power in control conditions for the eight slices tested. Error bars: SEM Reduction in the power spectrum from 50 Hz to 2050 Hz: 49.14% ± 45.48; *p < 0.05; Kolmogorov-Smirnov test; *n* = 8 cells; 10 recordings per cell. **(I)** Black: extracellular recording a pyramidal neuron from the subiculum recorded in low Mg^2+^. Orange: mibefradil (16 μM). **(J)** Time-frequency spectrograms of recurrent bursts. **(K)** Mean summed power spectrum analysis of recurrent bursts of the slice in **(I,J)**. Error bars: SD Kolmogorov-Smirnov test; *n* = 10 sweeps. **(L)** Mean summed power spectrum of recurrent bursts in mibefradil as a function of the mean summed power in control conditions (*n* = 6 slices). Error bars: SEM Reduction in power spectrum from 50 Hz to 2050 Hz: 82.8% ± 30.7; Kolmogorov-Smirnov test; *n* = 6 cells, 10 recordings per cell. **(M)** Black: extracellular recording a pyramidal neuron after removal of extracellular Mg^2+^. Blue: recording from the same cell in the presence of DOI (10–50 μM). Scale bars: 20 mV and 100 ms. **(N)** Time-frequency spectrograms of recurrent burst in control condition and in the presence of DOI. **(O)** Mean summed power spectrum analysis of recurrent bursts of the slice illustrated in **(M,N)**. Error bars: SD Kolmogorov-Smirnov test; *n* = 10 sweeps. **(P)** Mean summed power spectrum of recurrent bursts in DOI as a function of the mean summed power in control conditions for the eight slices tested. Error bars: SEM Reduction in the power spectrum from 50 Hz to 2050 Hz of 30.9% ± 41.5%, Kolmogorov-Smirnov test (*n* = 6 cells with 10 recordings from each cell). **(Q)** Example of cell-attached recording of spontaneous seizure-like activity in the subiculum in the absence of extracellular Mg^2+^. ^*^p < 0.05; ^*^^*^p < 0.01; ^*^^*^^*^p < 0.001.

Since bursting neurons initiate epileptiform activity in the subiculum (Harris and Stewart, 2001a; Cohen et al., 2002; Menendez de la Prida and Gal, 2004), we tested the effect of the T-type Ca^2+^ channel blocker mibefradil in slices with epileptiform activity induced by low extracellular Mg^2+^ concentration. Mibefradil strongly decreased the occurrence of epileptiform discharges evoked in the subiculum by stimulation of CA1 in all slices tested (Figures 4I–L).

Finally, we tested the effect of a 5-HT_2_ receptor agonist on seizures evoked by electrical stimulation of the CA1 region in slices where epileptiform activity was induced by lowering the extracellular concentration of Mg^2+^ ions. Bath application of the 5-HT_2A/2C_ agonist DOI hydrochloride significantly decreased the intensity of epileptiform discharges evoked in the subiculum (Figures 4M–P).

## Discussion

Our results show that 5-HT exerts a powerful inhibitory control of the excitability of principal cells from the subiculum by inhibiting their bursting behavior. By activating 5-HT_2C_ receptors, 5-HT selectively inhibits the T-type Ca^2+^ channels responsible for the burst. In addition to the inhibition of bursts, we found that 5-HT hyperpolarized the membrane of principal cells from the subiculum. This latter effect resembles the hyperpolarization caused by the activation of 5-HT_1A_ receptors in CA1 pyramidal cells (Andrade and Nicoll, 1987). However, the amplitude and the duration hyperpolarization induced by 5-HT (Figure 1D) were comparable to the ones induced by agonists for 5-HT_2C_ receptors (Figure 3B), suggesting that most of the effect was caused by 5-HT_2C_ receptor activation, even though we cannot exclude the involvement of other serotonergic receptors. Since most of the hyperpolarization was inhibited by relatively low concentrations of mibefradil (Figures 2E,F), we concluded that it originated from the inhibition of a window T-current present at rest (Figure 1B). Blocking T-type Ca^2+^ channels also produces a hyperpolarization of thalamic neurons of 1–2 mV (Dreyfus et al., 2010) comparable to the one reported here (Figures 2E,F). Such window currents indicate that bursts can be evoked from resting membrane potential.

### Pathway Responsible for the Inhibition

5-HT_2C_ receptors are coupled to G proteins consisting of G_αq_ and G_βγ_ complex. G_α_ induces phospholipase C (PLC) to hydrolyze phosphatidylinositol 4,5-bisphosphate (PIP_2_) to inositol 1,4,5-triphosphate (IP_3_) and diacyglycerol (dAG). IP_3_ triggers the release of Ca^2+^ from intracellular stores, which, together with dAG, activates protein kinase C (PKC). The activation of G_αq_ coupled receptors has been reported to inhibit Ca_V_3 channels. In heterologous systems the G_αq_ coupled neurokinin 1 receptor induces the inhibition of recombinant Ca_V_3.2 channels via a pathway that involves G_αq_, PLC, and PKC (Rangel et al., 2010). In contrast, the G_αq_ coupled dopamine D1 receptor expressed in adrenocarcinomal cell line H295R inhibits Ca_V_3.2 channels via the G_βγ_ complex that binds to an intracellular loop of the Ca^2+^ channel (Wolfe et al., 2003). More experiments will be required for determining if the inhibitory pathway we uncovered in the subiculum involved any of these two molecular mechanisms.

### Physiological Relevance

The modulatory pathway we uncovered could have profound effects for spike-timing-dependent plasticity in the subiculum. It was recently shown that the coincidence of bursts with excitatory synaptic inputs triggers LTD of synaptic transmission (Pandey and Sikdar, 2014). In contrast, when bursts are anti-causally paired with excitatory synaptic inputs, LTP is promoted. The selective inhibition of bursts could therefore inhibit LTD or LTP, depending on the relative timing of synaptic input and bursts. In addition to glutamate, subicular neurons express neurotensin (Roberts et al., 1984). The release of neuropeptides occurs only during high frequency discharge of presynaptic neurons (Bloom et al., 1987). In agreement, it was shown that mesocortical neurons release neurotensin during bursts but not during low frequency firing (Bean and Roth, 1991). By inhibiting the burst firing, 5-HT could therefore primarily prevent the release of neurotensin without affecting the release of glutamate.

### Antiepileptic Effect of Serotonin

Our data show that the activation of 5-HT_2C_ receptors decreases the occurrence of epileptiform discharges in the subiculum by inhibiting T-type Ca^2+^ channels responsible for the epileptic behavior of the temporal lobe (Yaari et al., 2007). By linking 5-HT receptors and T-type Ca^2+^ channels, we have uncovered a mechanism that unifies aspects of the pathology that until now were considered separately. TLE usually arises in the subiculum (Behr and Heinemann, 1996b; Harris and Stewart, 2001b; Cohen et al., 2002; Wellmer et al., 2002; Cavazos et al., 2004; Menendez de la Prida and Gal, 2004; Stafstrom, 2005; Wozny et al., 2005; Knopp et al., 2008).

Several observations indicate that 5-HT reduces the susceptibility to seizures occurring in TLE. An increase in concentration of 5-HT induced by blocking its reuptake from the extracellular space decreases the number of seizures (Prendiville and Gale, 1993; Yan et al., 1994; Bagdy et al., 2007; Buchanan et al., 2014). Conversely, drugs that decrease the concentration of 5-HT in the brain promote seizures in animal models of epilepsy (Wenger et al., 1973; Maynert et al., 1975; Lazarova et al., 1983), while knocking-out the gene encoding for 5-HT_2C_ receptors facilitates epileptic seizures (Tecott et al., 1995; Applegate and Tecott, 1998; Upton et al., 1998). In addition, the 5HT_2C_ agonist 3-Trifluoromethylphenylpiperazine (TFMPP) reduces spontaneous seizure activity in the pilocarpine model of TLE (Hernandez et al., 2002).

One of the long-term changes associated with mesial TLE is a strong increase in the proportion of bursting cells in the subiculum (Faas et al., 1996; Su et al., 2002; Wellmer et al., 2002; Yaari et al., 2007; Becker et al., 2008). Two strong arguments suggest a link of causality between T-type Ca^2+^ channels and TLE. First, epileptic seizures are initiated by bursting neurons in subiculum (Harris and Stewart, 2001a; Cohen et al., 2002; Menendez de la Prida and Gal, 2004). Second, after status epilepticus, regular firing hippocampal neurons acquire burst-firing properties caused by an upregulation of the T-current (Su et al., 2002). Serotonergic fibers projecting to the hippocampus originate mainly from the median raphe nucleus (Azmitia and Segal, 1978). They are characterized by a spontaneous regular discharge of action potentials (Jacobs and Azmitia, 1992) suggesting tonic release of 5-HT in the hippocampus. This release may prevent the occurrence of seizures under physiological conditions.

Both antiepileptic (Prendiville and Gale, 1993; Yan et al., 1994; Bagdy et al., 2007; Trivedi and Kurian, 2007; Buchanan et al., 2014) and proconvulsive (Rosenstein et al., 1993; Pisani et al., 1999; Trivedi and Kurian, 2007) effects induced by antidepressors acting on the serotonergic system have been reported. How does this fit with our findings? A systematic review of the literature shows that the proconvulsive effects are induced by tetracyclic antidepressants such as Maprotiline or Amoxapine (Pisani et al., 1999) and tricyclic antidepressants such as Imipramine (Rosenstein et al., 1993). These molecules have high affinity for other targets such as norepinephrine transporter, alpha-1 adrenergic, histamine or muscarinic receptors and it is likely that their pro-convulsant activity is due to these latter actions (Montgomery, 2005). In contrast, selective serotonin re-uptake inhibitors (SSRIs) act specifically on 5-HT transporters. When tested on epileptic patients, they do not promote seizures more than placebos (Rosenstein et al., 1993; Pisani et al., 1999; Montgomery, 2005) but on the contrary decrease their occurrence (Favale et al., 1995, 2003; Kondziella and Asztely, 2009). Our results are therefore not in contradiction with the consensus that SSRIs do not significantly increase seizure frequency in epileptic patients (Trivedi and Kurian, 2007).

Our data suggest that the antiepileptic effect of 5-HT is caused by the selective inhibition of T-type Ca^2+^ channels. Different drugs such as Zonisamide or Trimethadione, acting as T-type channels blockers are commonly used for treating absence seizures. They have also proven to be efficient on several animal models of TLE (Löscher, 2002) as well as for patients suffering from partial and generalized epilepsy (Lancaster, 1980; Shorvon, 2010; Holder and Wilfong, 2011). By linking 5-HT receptors and T-type Ca^2+^ channels, we have uncovered a mechanism that unifies aspects of the pathology that until now were considered separately. The physiological mechanism might be used as a new strategy for treating TLE patients and people with a high risk of developing TLE such as children with febrile seizures (Patterson et al., 2014).

## Author Contributions

AVP and J-FP designed and conceived the experiments. AVP performed the electrophysiology experiments. CSJ and AVP performed the immunohistochemical stainings. J-FP supervised all the experiments. VC co-supervised the experiments on pilocarpine treated animals. AVP and J-FP wrote and prepared the manuscript. All authors reviewed the manuscript.

## Conflict of Interest Statement

The authors declare that the research was conducted in the absence of any commercial or financial relationships that could be construed as a potential conflict of interest.
